The article "An Intelligent Recommendation Method for Tourist Attractions Based on Deep Learning" was published in 2022. Journal: Comput Intell Neurosci.

# An Intelligent Recommendation Method for Tourist Attractions Based on Deep Learning

**DOI:** 10.1155/2022/3974109

**Published:** 2022-05-18

**Authors:** Manhua Yang

**Affiliations:** College of Agriculture and Bioengineering, Taizhou Vocational College of Science & Technology, Taizhou 318020, Zhejiang, China

## Abstract

Tourists are the people who can be seen all over the world. Therefore, this has increased the demand for product supply in tourist locations. Technological development would be the only solution to solve those issues related to the demand and supply of the products. Furthermore, a tourist needs enough information about the country he wishes to travel. Some specific data required include hotels, destinations, malls, and tourist places, and they are needed before they land on the tourist country. The data collection can be achieved by applying trending technologies such as deep learning algorithms and some intelligent systems. Furthermore, the tourist may collect information about the locations through feasible devices such as laptops and mobile phones. Among the varying devices and technologies, the most preferred and convenient device should be carried wherever they travel with ease. For example, cellular phones may be considered the easiest modem to carry and use with this specification. In this perspective, the lightweight deep learning model will make significant technology access to resources. Typically, deep learning models are designed with the prospect of extracting the features, potentially to create easy tool access within the mobile accessing service. Visual Bayesian Personalized Ranking (VBPR) Algorithm using DL is implemented for initiating the recommendation system for tourist attractions in any given location. The proposed model was compared with various existing algorithms, and it was found that the proposed system had delivered 98.56% of accurate recommendations for tourist travelers.

## 1. Introduction

Traveling throughout the world has never been easier than it is now, with the development of the availability of online travel booking websites. The amount of information available on the Internet grows exponentially, and travelers have more difficulty locating what they are looking for [1]. A significant reduction in the problem of data overflow has occurred due to the use of recommendation algorithms. A website platform analyses the user's explicit and implicit information to select the most appropriate products. Many algorithms have been developed to understand the overall system [2] better. Because of the substantially different illumination conditions between night and day, developing a nighttime travel suggestion system has proven to be difficult [3]. However, there are more effective suggestions depending exclusively on daytime travel statistics. This work demonstrates that an issue can be solved by utilising novel image processing approaches. On the one hand, image processing frequently overlooks the underlying reasons for image degradation [4]. Instead, specific approaches are employed to increase the visual impact of an image and make it easier for people or computers to analyze or interpret an image, among other things. Ultimately, the essential purpose of an image is to communicate an idea to the viewer visually. For example, when it comes to image enhancement, there are two sorts of approaches: spatial domain and frequency domain [5]. The term “spatial-domain” refers to gray-value arithmetic processing in the spatial domain. Color processing and grayscale transformations are two examples of these modifications to the software. On the other hand, an improved image is produced when the frequency domain technique is used, which results from a more excellent transform value [6].

It is recommended that collaborative filtering (CF) techniques be used to recommend items. Almost all of them are employed in some capacity regularly. The past content consumption is used to make product recommendations based on interest models [7]. The system only generates a small number of recommendations, a significant shortcoming. This information can be used to identify individuals who share similar interests, allowing for more focused recommendations to be made for them. While it is theoretically possible for a hybrid recommendation algorithm to correct the shortcomings of earlier algorithms, constructing such an algorithm is more challenging than developing the others [8]. This study focused on evaluating the tourists attractions using deep learning.

## 2. Related Work

There has been a significant advancement in artificial intelligence in the last few years. In recent years, deep learning has developed as a critical component of many firms' artificial intelligence strategies. Deep learning can be used in image, text, and natural language processing to mine data features for confidential information that is otherwise difficult to detect [9]. For example, visitors and the regions they traveled were once used to selecting which picturesque spots to visit, rather than considering the travelers' traits. Feature representations between different video input formats can be created to extract additional information from video data [10]. For example, a recursive neural network suggested new movies based on user and movie time series data. It is feasible to improve the accuracy of suggestions by making use of both long-term and short-term memory units at the same time. Many recommendation systems combine user feedback with images of well-lit tourist attractions, routinely used as input [11]. For some, nighttime travel is more popular than daytime travel vacation. One of the most challenging aspects of this research has been figuring out how to deliver safe evening driving directions in dimly lit areas. This article generates travel ideas at night by combining a convolutional neural network and a night image enhancement method based on histogram equalisation, among other techniques [12].

One of the most crucial considerations is seeing and doing when planning a vacation. For tourists, cities worldwide provide many things to see and do [13]. It is nearly impossible to generalise cities because they all have distinct characteristics that cannot be generalised. With so many options available, travelers can find it difficult to choose locations that meet their needs and expectations. A tourist may become overwhelmed by the sheer number of things to see and do in a specific city when visiting it for the first time [14]. Using a trip recommendation system can help you save both time and money on your travels. In order to put a recommendation system in place, there are several options. These systems were popular in the past, including recommender systems that combine content-based and collaborative filtering, becoming increasingly popular [15]. In the context of collaborative filtering, the term “neighborhood” refers to a group of people who have similar profiles and interests and who are working together to solve a problem. By its parameters and the information provided by the user, the system generates recommendations for the user [16]. People are more inclined to be interested in things they have already rated or viewed, so content-based tactics are used to attract their attention. With this content-based strategy, you may identify and target consumers based on their previous purchases [17]. Alternatively, it is feasible that a cold-start suggestion engine will not determine whether or not rating data has previously been collected. Images from previous travels might be utilised to produce recommendations for tourist attractions. According to the researcher, customers may prefer to communicate their preferences through visual cues such as images rather than verbal cues [18]. Recently, there has been much interest in the recommendation systems for tourist locations. Using social networking sites such as Facebook, Twitter, and Foursquare, creating a custom recommendation system for tourist destinations is possible. If the recommended system is experiencing difficulties, this process may restore it to full operation [19]. A growing number of companies are using deep learning to improve their recommendation systems. While the site was advertising Google Play, the site's architecture underwent a significant transformation. Deep learning was employed in order to produce movie recommendations [20]. The RNN-based algorithm used to produce the news suggestions was also used to generate the recommendations. It was possible to develop a novel content-based method through the use of deep belief networks and probabilistic graphical models. Several studies have found that deep learning recommendation systems outperform those based on more traditional methods. Due to the increase in the number of people who use smartphones, academic interest is increased in developing innovative ways to incorporate recommendation algorithms into mobile applications [21]. An ontology-based hybrid recommendation technique has been created and tested to recommend museums based on the user's query and location. Customers were able to determine the most efficient route between two points using knowledge-based recommender systems and group filtering techniques. An individual's mobile phone's RSS (received signal strength) could be exploited to get beyond GPS and RFID constraints. The capacity of this system to make recommendations and attract new users has been proven through the usage of RSS feeds and user preferences [22]. This contextually aware and knowledge-based technology may generate movie recommendations for you based on your geographic location and previous viewing patterns, among other factors. The number of people that participated, the time of day, and the user's geographic location were all taken into consideration when generating the results. Taxi drivers may use a smartphone recommendation system to discover the most convenient pick-up spots. This research focuses on developing an image-based tourism recommendation system [23]. Images of prominent holiday destinations can be obtained using an image search or through a user's previous trip photos. Deep learning is used to classify pictures, which allows for more accurate classification. By comparing two sets of photos side by side, it is possible to determine whether or not they are sufficiently comparable. The tourist sites and activities in Yogyakarta serve as case studies for our investigation (Indonesia). As a result of this new strategy, visitors may expect more precise information about where and when to travel on their next trip. Today, it is the most widely recognised type of architecture globally [24]. The Efficient Net and Efficient Net-Lite edge architectures were utilised to develop a deep learning recommendation model using deep learning. Using the Efficient Net approach, Efficient Net beats current CNNs by 8.4x and 6.1x on the Image Net dataset, respectively. Among the many tasks that may be completed with effective Internet technology is image and speech recognition and video identification and verification. An efficient net makes predicting and recognising trends easier by reducing their complexity [25]. In addition, Efficient Net points out that it can manage huge files on mobile devices as well. The Efficient Net-Lite architecture is employed in the recommendation system for tourists developed by our research team.

### 2.1. Motivation for the Study

It comprehensively examines and analyses massive tourist attraction image extractions, utilising multiple linear regression algorithms. This method typically relies on grid partitioning, which is helpful in finding that the overall similarity of distinct images is high. The Business Oriented Framework (BOF) method is represented by the information extraction method, which generally retrieves the image's local features. These features use the structurally complex assist in addressing, cluster the others using Visual Bayesian Personalized Ranking (VBPR) to produce a small visual glossary, and categorise the feature representations using a graph variable related to the visual schema. However, if there are many different images, the dimension of a visual vocabulary will be significant, making the development of the BOF model challenging. The image characteristic is chosen as the last fully connected layer, which utilises the principal components approach. Then, the slight characteristic is organised and constructed solely using DL's VBPR Algorithm. Our network retrieval efficiency has increased by 98.43% with the utilisation of deep neural networks to extract features and the high efficiency of a hash data set for retrieval. These are used to overcome the shortcomings of the control list in accuracy and some other aspects of image search. A BOF model—a business model framework seems to be a theory-dependent description of a firm, its internal processes, and its connections—is frequently defined as a normative statement on what should be included in it.

## 3. Materials and Methods

Here the entire development application is managed with the power of an algorithm, which is TensorFlow Lite. It is one of the frameworks that are stored behind the coding knowledge of machine learning and artificial intelligence, and here it is being collaborated with to form a new technology that helps tourists. With the help of the TensorFlow Lite framework, it is possible to create a lightweight solution for both mobile and embedded devices. It establishes a clear relationship between the acceptance of machine learning concepts in mobile devices and the acceptance of machine learning concepts in general through this concept. Consuming reduced latency flow is an advantage for further classification or making important things with regression, etc. This framework algorithm creates a field that an application can access without incurring round trips to the server. Like the C++ and Java wrappers, the application is maintained behind the mobility service. Other than this segment, as an Android user, there would be a neural networking API that focuses on the development of hardware acceleration. However, here, the problem is that it is harder to use this kind of framework without developing a trained model. For the first time, it is asked to prepare the trained model with the help of a high-powered machine. Once the process is completed by creating a separate model, then it can be started for the further procedure to implement the model into a TensorFlow Lite framework. This framework is depicted in Figure 1.

In recent days, more than Google Maps, social media has become one of the fastest distributed and most used applications. According to the author, here, the author has worked on the concepts by integrating the intelligence method by gathering such information from Twitter and other social media development applications. Computational intelligence has significant future growth potential, and advancements in deep learning platforms are increasing by incorporating multiple data files into the machines. To further develop and overcome the issues, making changes in architecture and initialising some parameters behind the deep learning models are essential. At the same time, implementing such an application in a lightweight model is also a challenging problem. Most multinational companies are building their ML libraries to make things automated. In another case, making suggestions through past travel images, videos, and audio files stored on social media would recommend a perfect experience model to create a better deep learning technology. According to the world population, mobile users are at their maximum compared to laptops and other device users. In that case, creating software adaptable to mobile devices would increase the number of users. While testing this algorithm, the accuracy of the result is about 85%, where the average score equals 4.1. To examine the working process of deep learning models, Google Translate can be taken as one of the best examples; if an enormous paragraph is to be converted to another language within a fraction of a second, the search engine is ready to show its result with 90% accuracy. This is how the deep learning module functions with real-time applications. Not only the translating site, but also the gallery maintenance and other gatherings are only possible with the help of a deep learning algorithm.

A tourist must have sufficient knowledge of the nation to which he desires to go. Hotels, destinations, malls, and tourist destinations and before they land in the tourist country are some of the specific details necessary. Data collecting may be accomplished through the use of trending technology such as deep learning algorithms. Tourists can gather information about the destinations using portable equipment such as laptop computers and cell phones. The lightweight deep learning model will increase technological access to resources significantly. Deep learning models are often created with the goal of extracting features and maybe creating quick tool access inside the mobile accessing service. A Visual Bayesian Personalized Ranking (VBPR) Algorithm based on deep learning (DL) is used to initialise the recommendation system for tourism attractions in each given region. The multiprocessor learning method is represented by *ab* to build a Visual Bayesian Personalized Ranking (VBPR) and *U*^*R*^ defines a classification method of integrated modules that would be launched within the VBPR framework. In particular, this research would discuss the *d* graph's creation using BOF method and the associated optimisation method based on semisupervised multiprocessing learning.

(1) $$\begin{array}{c} \partial_{1}d^{2}\leq \int_{r_{0}}^{r_{0}+R_{0}}{\left|U^{R}\left(\tau \right)d\right|}^{2}ab\left(\tau \right)\leq \partial_{2}d^{2},\;\forall_{r0}\geq 0,\;r\in C^{p}. \end{array}$$

*τ* denotes to classify the complexity of calculation represented in multiprocessor integrated to grows considerably  *∂*_1_*d*^2^ (refer to (1)) as the structures lengthen all through this probability computation approach. The parameters of the model |*U*^*R*^(*τ*)*d*|^2^*ab*(*τ*) ≤ *∂*_2_*d*^2^,  ∀_*r*0_ ≥ 0 are practically hard to *C*^*p*^ estimate on present hardware. The presence or absence of  *f*^*p*^(*r*) in such a sentence is exclusively decided by the *r* term preceding its framework and is given in

(2) $$\begin{array}{c} f^{p}\left(r\right)=\underset{g⟶0}{\lim}\frac{1}{g^{p}}\sum_{q=0}^{p}{\left(-1\right)}^{q}\left(\begin{array}{c} p\\ q \end{array}\right)f\left(r-qg\right). \end{array}$$

A *p*, *q* sentence's similarity is measured exclusively by −sent(∇^*a*^*x*/|∇^*a*^*x*|+*t*) the two or more words before the framework and is defined in

(3) $$\begin{array}{c} -\text{sent}\left(\frac{\nabla^{a}x}{\left|\nabla^{a}x\right|+t}\right)+\lambda_{e}\left(x-x^{0}\right)=0, \end{array}$$

*q*_*i*_(*h*) of (4) is the students' linguistic *h*  level that aims to represent the distinction between both the learners *x* cognitive stage and the difficulty level to learning resources.

(4) $$\begin{array}{c} q_{i}\left(h\right)=\frac{f_{i}r_{i}-\text{bad}\left(h\right)}{\text{good}\left(h\right)-\text{bad}\left(h\right)}. \end{array}$$

The learner's progression is indicated by *E*_*i*_^*n*^(*r*), the distinction of which lets the viewer realise *h* encompassed within learning material and also the information notes the student wants to acquire. The smaller the difference, the more closely *n* training resource's expert values match randam_*j*_*E*_*ij*_^*n*^(*r*); the driver's license information points are depicted in

(5) $$\begin{array}{c} E_{i}^{n}\left(r\right)=\sum_{j\in L}{\text{randam}}_{j}E_{ij}^{n}\left(r\right). \end{array}$$

(*u*, *w*; *A*, *ϕ*) of (6) presents the optimisation technique of spending, while the instructional content represents the whole spending data among training resources.

(6) $$\begin{array}{c} \left(u,w;A,\phi \right)={\left|d\right|}^{-0.6}\int_{-\infty }^{+\infty }d\left(\tau \right)h\left(\tau -r\right)e^{-jb\tau }\text{d}\tau . \end{array}$$

*b*_*i*_ is the fundamental requirement for the given period of education *L*_*pp*_(*u*) (refer to (7)) and it represents the objective that emphasises the different learning time required to complete teaching programs  *b*_*i*_*U*_*i*_(*u*)=*B*^*R*^*U*(*u*) with learning time consumption.

(7) $$\begin{array}{c} L_{pp}\left(u\right)=\sum_{i=1}^{P}b_{i}U_{i}\left(u\right)\\ =B^{R}U\left(u\right). \end{array}$$

The driver's license is utilised to calculate the total optimisation performance and is given by  *ϕ*_*q*,*p*_. The learning route is established by the comments thread function through recalibrating coefficients; as indicated by (8), it is a functional demonstration of the personalised learning path optimisation approach.

(8) $$\begin{array}{c} \phi_{q,p}=\frac{Q_{q,p}^{2}}{\delta^{2}}\exp\;s\left(\frac{\left(Q_{q,p}*A\right)}{3\delta^{2}}\right)*\left[e^{i\left(Q_{q,p}*A\right)}-e^{-\delta^{2}/3}\right]. \end{array}$$

In the algorithm, *φ* divides the confirmation e-mail of a particle's propagation direction into three phases: speed opposition, self-learning, and social behaviour. The ∑_*i*=1_^*O*^*Q*_*i*_*P*/*U*(*Q*_*i*_ ∈ *Q*) stance updating of a material with and in generation has indeed been determined by a particle's stance *t* formation but also the generation needs motion orientation, as explained in

(9) $$\begin{array}{c} e=\frac{{\left(\varphi \phi_{35}+\varphi \phi_{04}\right)}^{2}+4\varphi \phi_{22}^{2}}{{\left(\varphi \phi_{35}+\varphi \phi_{04}\right)}^{2}}, \end{array}$$

(10) $$\begin{array}{c} B=\frac{\sum_{i=1}^{O}Q_{i}P}{\sum_{i=1}^{O}P_{i}} \end{array}$$

A tourist must have sufficient knowledge of the nation to which he desires to go: hotels, destinations, malls, and tourist destinations and before they land in the tourist country are some of the specific details necessary. The state of the *∂K*/*∂u* particle has already been defined from the aspect of  *Q*″ possibilities. Each particle's *q* ^″^ bit value in domain is 0 or 1, and the equation is exactly as explained in

(11) $$\begin{array}{c} Q{\;}^{\prime \prime }=\left\{Q{\;}^{\prime \prime }|q{\;}^{\prime \prime }=\frac{q{\;}^{\prime }\times n}{N},\forall q{\;}^{\prime }\in Q{\;}^{\prime }\right\}, \end{array}$$

(12) $$\begin{array}{c} \frac{\partial K}{\partial u}=\sum_{i=1}^{p}\left[h_{i}-\frac{\exp\;s\left(u+\sum_{j=1}^{q}u_{ij}\beta_{j}\right)}{1+\exp\;s\left(u+\sum_{j=1}^{m}u_{ij}\beta_{j}\right)}\right]=0. \end{array}$$

A machine learning representation is a representation where each texture relates a transformation technique to the surface *T* ∈ *S*^*N* ×*D*^ preceding it, referred to as no transformation to an edge before it. *M*^*p*^ ∈ *S*^*d*_*p*−1 × *d*_*p*__^ to achieve a  *d*_*p*_ directional recognition *p* − 1,  *T*_*p*−1_ ∈  *S*^*N*×*d*_*p*−1_^ a matrix able to represent a linear transformation applicable to a layer *p* − 1 production to receive a  *d*_*p*_ dimensional recognition *T*_*p*−1_*M*^*p*^ ∈ *S*^*N*×*d*_*p*_^ .

A deep learning representation is a representation, and each texturing relates a wavelet transform to the surface *T* ∈ *S*^*N*×*D*^ preceding it, also known as no modification to an edge before it. *M*^*p*^ ∈ *S*^*d*_*p*−1 × *d*_*p*__^ to achieve a *d*_*p*_ direction recognition *p* − 1, *T*_*p*−1_ ∈  *S*^*N*×*d*_*p*−1_^ a matrix capable of representing a transform applicable to the a layer *p* − 1 generation to receive a *d*_*p*_ dimensional *T*_*p*−1_*M*^*p*^ ∈ *S*^*N*×*d*_*p*_^.

(13) $$\begin{array}{c} T\in S^{N\;\times D}=\sum \psi \left(T,M^{1},\ldots ,M^{k}\right)+M^{p}\in S^{d_{p-1\times d_{p}}}\;\\ =\psi_{K}\left(\psi_{K-1}\left(\ldots \psi_{2}\left(\psi_{1}\left(TM^{1}\right)M^{2}\right)\ldots M^{p-1}\right)M^{p}\right)+\;T_{p-1}M^{p}\in S^{N\times d_{p}}. \end{array}$$

This should be emphasised as *A*  ×  *B* matrix, where *B* = *d*_*p*_ seems to be the component of the network's input that corresponds to the number of categories with a certain case of a classification algorithm.

(14) $$\begin{array}{c} B=d_{p}=A\times B\int \underset{{\left\{M^{p}\right\}}_{p=1}^{P}}{\min}l,\;\Phi \left(H,M^{1},\ldots ,M^{P}\right)+\lambda \Theta \left(M^{1},\ldots ,M^{p}\right)p-1,\;T_{p-1}\in S^{N\times d_{p-1}}, \end{array}$$

where  *h*_*i*_(*T*) describes a standard set of viable stem discipline in reaction to producing precise *X* in an infinite dimensional space  *h*_*i*_(*T*) ∈ *V* between all concealed alternate machine kernel functions.

(15) $$\begin{array}{c} h_{i}\left(T\right)=\sum T_{p-1}M^{p}\in S^{N\times d_{p}}+\sum_{i=1}^{T}{\left\{T_{i}\in D^{2}\left(\Omega \right),H_{i}=f\left(T_{i}\right)\right\}}_{i\in I}. \end{array}$$

As a consequence, deep learning algorithms use typically distributed data and prediction to local transcriptions. A VBPR is made up of many deep convolutional networks of the kind *T* = BM (T), which act on the a p-dimensional output *T*(*u*)=(*T*_1_(*u*),…, *T*_*p*_(*u*)) by using a filtration institution and also argument multivariance *ψ*.

(16) $$\begin{array}{c} \tilde{T_{l}}\left(u\right)=BM\left(T\right)+\psi \left(\sum_{p=1}^{P}\left(T_{l}*wl\cdot v\right)\left(u\right)\right)-T\left(u\right)\\ =\left(T_{1}\left(u\right),\ldots ,T_{p}\left(u\right)\right). \end{array}$$

Generating a q-dimensional outcome *T*(*u*)=(*T*_1_(*u*),…, *T*_*q*_(*u*)) is another possible term for features extracted. Eventually,

(17) $$\begin{array}{c} \left(T*w\right)\left(u\right)=\int_{\Omega }T\left(u-u{\;}^{\prime }\right)w\left(u{\;}^{\prime }\right)\text{d}u{\;}^{\prime }+\int T\left(u\right)=\left(T_{1}\left(u\right),\ldots ,T_{q}\left(u\right)\right). \end{array}$$

The classical translation function is represented by this symbol. The filter *Z* has reduced spatial support, according the deflection before. $\tilde{T_{l}}\left(u\right)$ is an up-testing technique or convolution that can be employed.

(18) $$\begin{array}{c} \tilde{T_{l}}\left(u\right)=Z\left(\left\{T_{l}\left(u{\;}^{\prime }\right):u{\;}^{\prime }\in N\left(u\right)\right\}\right),\;l=1,\ldots q. \end{array}$$

## 4. Results and Discussion

The data displayed on the result in Figure 2 is that the mobile node is done through the various mobile result that displays the module, along with the destination tourist guide module. The results display component for mobile terminals contains general information about just the attractions introduced through the attraction tourist guide module, which provides further data about the destination, like the humanities and adjacent commercial information. A grayscale founder matrix is used in this paper chosen and added.

The complexity of the calculation grows considerably  *∂*_1_*d*^2^ as the structures lengthen all through this probability computation approach. The parameters of the model |*U*^*R*^(*τ*)*d*|^2^*ab*(*τ*) ≤ *∂*_2_*d*^2^, ∀_*r*0_ ≥ 0  are practically hard to estimate on present hardware. The presence or absence of  *f*^*p*^(*r*) in such a sentence is exclusively decided by the term preceding its framework of an image's colour and light. Figure 2 shows the intensity. For the result analysis for feature map (refer to Table 1), the mixture approach determines the relationship here between Mobile GPS collection and images with tourist guide of scenic spots grayscale within every direction image and across various pixels and represents the geographical distribution.

The very first classification of photos based on texture dispersion and picture complexity is given in Figure 3. This dissertation separates the original data into different subsets when utilising correlation to categorisation, and then, after numerous data tests, the specific value difficulties that potentially split the subgroups have been identified. A spectrum of computations is created after analysing all of the picture correlation values, and three values should be established in order to categorise those subgroups. To simplify data statistics, a number higher than just a certain quantity is used for comparisons, and the pixel values collected include 550, 1100, and 1450, and also the equal instances are separated into another statistical subgroup. Depending on this, a further division is done using the same manner as before, and also the final spectrum is determined through ongoing experimentation with various values. The test results on the picture set were also quite precise. Because the relationship similarity is measured exclusively by −sent(∇^*a*^*x*/|∇^*a*^*x*|+*t*), the two or more words before the framework are shown in Figure 3. 1101 photos met required connection with such a values higher than 0.166, completing the separation of two categories. 1451 pictures are obtained with values larger than 0.086. Ultimately, four groups of 550 photos each could be obtained, and trials on large data can produce even excellent performance. Result analysis for multiple linear regression training and testing performance in tourist attractions based on deep learning is shown in Table 2.

After analysing all of the picture correlation values, a spectrum of computations is created, and three values should be established to categorise those subgroups. To make data statistics easier to understand, a number greater than a specific quantity is used for comparisons, and the pixel values collected are 550, 1100, and 1450, with equal instances separated into a separate statistical subgroup. Using the same method as before, a further division is made, and the final spectrum is determined through ongoing experimentation with various values. Because the relationship similarity is measured exclusively by the two or more words before the framework, the test results on the picture set were also quite precise. In the training and testing for the GPS methodology (89.67%) for collection of mobile images (91.56%) in tourist guide to picturesque locations (90.67%) for extraction of mobile features (94.23%), analysis for multiple linear regression training and testing performance in tourist attractions based on deep learning is shown in Table 2.

In massive tourist attraction feature extraction, we must query the consistency and validity of individual attractions in order to determine the average consistency and validity of many attractions. It is being used to describe the general effectiveness of user query and then provide 30 photos that are comparable to each attraction by frequency on similarity from a sum of 500,000 images of 1740 sights online; request 1000, 2000, 5000, and 7000, but also 10000 attractions, including both; but also determine the mean accuracy and average comprehensiveness of the retrieved documents belonging to a queried theme parks. Texturing relates a wavelet transform to the surface *T* ∈ *S*^*N* ×*D*^ preceding it, also known as no modification to an edge before it. *M*^*p*^ ∈ *S*^*d*_*p*−1 × *d*_*p*__^ to achieve a *d*_*p* _ direction recognition *p* − 1,  *T*_*p*−1_ ∈  *S*^*N*×*d*_*p*−1_^, a matrix capable of representing a transform applicable to the a layer *p* − 1 generation to receive a *d*_*p* _ dimensional *T*_*p*−1_*M*^*p*^ ∈ *S*^*N*×*d*_*p*_^ as shown in Figure 4. According to Figure 4, also as quantity of query websites increases, the mean search accuracy overall completeness drops, owing to the varying data quantity of various sites inside the tourist attractions dataset and the different images within image dataset contributes to modest loss an accuracy. Though we can see the general drop in average accuracy and completeness also is not significant, we can conclude that the approach employed for huge tourist attraction picture retrieval is stable.

Figure 5 shows that the upgraded VBPR model's recall rate is much higher than the comparative background for almost the same reasons stated before. As the quantity of suggested attractions grows, the recall rate is less unstable than NMF among the KNN. This suggests that its upgraded VBPR method can be recommended in various attractions. Hybrid recommendation (HVM) fully utilises the user traveling information and recommended outcomes of the upgraded VBPR methods; also the recommended efficiency is ideal; that is, its user traveling preferences smooth out the final results shown above. The VBPR model seems to be the primary factor, with user travel choice information depending just on the stratified sample predictive method serving as an additional factor. The tourist attraction suggestion system based upon stratified sample statistics and an enhanced VBPR model may effectively increase recognition performance to match customer requirements to a more significant extent, relieving the information scalability issue. Moreover, the recommendations are more stable. Even though the enhanced VBPR model (see Table 3) can complete the recommendation, the visual features and also all impartial features are used, or the multimodal linguistic correlation among various image features is not adequately explored, but again recommendation effectiveness even now requires improvement.

## 5. Conclusions

Multiple linear regression algorithms were used to examine and analyse large-scale image extractions of tourist attractions. When the overall similarity of images is high, grid partitioning is a valuable technique. Using the BOF method, one can retrieve the image's local features that use the structurally complex assist in addressing, cluster the others to produce a small visual glossary, and categorise the feature representations using a graph variable related to the image's visual schema. However, the BOF model will be difficult to develop if there are many different images to be chosen using the Visual Bayesian Personalized Ranking (VBPR) Algorithm with Dynamic Linking (DL), and the slight characteristic is organised and constructed as the final fully connected layer, sufficient to use the principal components approach. Our network retrieval efficiency has risen by 98.43%. In order to overcome some of the shortcomings of the control list in image search, a deep neural network and a hash data set are used to extract features and retrieve data. In this research, multiprocessor learning method is not compared with VBPR and is considered to be implemented as the future enhancement.

## Figures and Tables

**Figure 1:** Advanced predictive model.

**Figure 2:** Intelligent recommendation feature map method for tourist attractions based on deep learning.

**Figure 3:** Intelligent recommendation for multiple linear regression performance in tourist attractions based on deep learning.

**Figure 4:** Average accuracy rate and average completeness rate intelligent recommendation method for tourist attractions based on deep learning.

**Figure 5:** Tourist attractions based on deep learning recall values for recommended systems are compared with huge tourist attractions visual filtering results.

**Table 1:** Result analysis for feature map.

Mobile GPS collection (%)	Collection of mobile images (%)	Tourist guide to picturesque locations (%)	Extraction of mobile features (%)
93.45	95.76	97.56	96.35

**Table 2:** Result analysis for multiple linear regression training and testing performance in tourist attractions based on deep learning.

Different methodologies	Distance (km)	Training/testing (%)	Accuracy (%)
GPS tracking on mobile devices	Based on the tourist attractions place	89.67	93.56
Collection of mobile images		91.56	95.34
Tourist guide to picturesque locations		90.67	96.89
Extraction of mobile features		94.23	98.33

**Table 3:** Comparison result analysis for existing method.

Algorithm	Training/testing	Accuracy
VBPR	97.45	98.56
IBCF	92.24	93.34
LBCF	90.24	91.42
HC	85.23	88.24
FCM	90.24	91.12
BPR	89.23	89.54
HVM	84.23	86.4

## Data Availability

The data used to support the ﬁndings of this study are available from the corresponding author upon request.
